# Enhanced IMP3 Expression Activates NF-кB Pathway and Promotes Renal Cell Carcinoma Progression

**DOI:** 10.1371/journal.pone.0124338

**Published:** 2015-04-28

**Authors:** Xuelian Pei, Muhan Li, Jun Zhan, Yu Yu, Xiaofan Wei, Lizhao Guan, Hakan Aydin, Paul Elson, Ming Zhou, Huiying He, Hongquan Zhang

**Affiliations:** 1 Key Laboratory of Carcinogenesis and Translational Research, Ministry of Education, and State Key Laboratory of Natural and Biomimetic Drugs, Peking University Health Science Center, Beijing, PR China; 2 Department of Pathology, Peking University Health Science Center, Beijing, PR China; 3 Department of Anatomy, Histology and Embryology, Peking University Health Science Center, Beijing, PR China; 4 Institute of Pathology and Laboratory Medicine, Cleveland Clinic, 9500 Euclid Avenue, Cleveland, Ohio, United States of America; 5 Department of Quantitative Health Sciences, Cleveland Clinic, 9500 Euclid Avenue, Cleveland, Ohio, United States of America; 6 Department of Histology and Embryology and Key Laboratory of Xinjiang Endemic and Ethnic Diseases, Ministry of Education, Shihezi University School of Medicine, Shihezi, Xinjiang, PR China; Peking University Cancer Hospital & Institute, CHINA

## Abstract

**Background:**

Insulin-like growth factor 2 mRNA binding protein 3 (IMP3) is expressed in metastatic and a subset of primary renal cell carcinoma (RCC). However, the role of IMP3 in RCC progression was poorly understood. We aim to uncover the mechanism of IMP3 in regulating clear cell RCC (CCRCC) progression and validate the prognostic significance of IMP3 in localized CCRCC.

**Methods:**

Caki-1 cells stably overexpressing IMP3 and Achn cells with knockdown of IMP3 were analyzed for cell migration and invasion by Transwell assay. RNA-seq was used to profile gene expression in IMP3-expressing Caki-1 cells. A cohort of 469 localized CCRCC patients were examined for IMP3 expression by immunohistochemistry using tumor tissue array.

**Results:**

IMP3 promoted Caki-1 cell migration and invasion, whereas knockdown of IMP3 by RNAi inhibited Achn cell migration and invasion. Enhanced IMP3 expression activated NF-кB pathway and through which, it functioned in promoting the RCC cell migration. IMP3 expression in localized CCRCC was found to be associated with higher nuclear grade, higher T stage, necrosis and sarcomatoid differentiation (*p*< 0.001). Enhanced IMP3 expression was correlated with shorter recurrence-free and overall survivals. Multivariable analysis validated IMP3 as an independent prognostic factor for localized CCRCC patients.

**Conclusion:**

IMP3 promotes RCC cell migration and invasion by activation of NF-кB pathway. IMP3 is validated to be an independent prognostic marker for localized CCRCC.

## Introduction

Renal cell carcinoma (RCC), now being the 6th leading cancer in men in the US, contributing to the estimated 63,920 newly diagnosed and 13,860 deaths from kidney cancer in 2014 [1]. In the recent decades, the incidence of RCC has been steadily rising by 2–4% each year. The incidence of RCC in Asia is lower than in US and Europe, while the mortality-to-incidence ratio is much higher in Asia than in the developed nations [2]. In China, limited studies showed there is obvious increment of the RCC morbidity in recent years with the increasing of early diagnosed cases. One-third of patients are diagnosed of RCC with synchronous metastasis and one-third of patients who have undergone surgical resection for local RCC will eventually recur and metastasize. The five years survival rate of the latter group is under 10%, even though the FDA recently approved new drugs targeting specific pathways (tyrosine-kinase inhibitors/mTOR-inhibitors),which is available for RCC [3]. The underlying mechanisms for RCC metastasis are still not fully understood and no molecular strategies are currently recommended for routine clinical use to improve risk stratification of patients with RCC. The most common histological type of RCC is the clear cell RCC (CCRCC), which represents approximately 80% of RCC [3]. Therefore, it is essential to develop prognostic biomarkers for localized CCRCC to offer possible personalized therapy.

IMP3 is a member of insulin-like growth factor 2 (IGF-2) mRNA- binding proteins (IMPs) family, consisting of IMP1, IMP2 and IMP3. IMPs bind to and influence the transportation, localization and stability of target mRNA, especially during early stages of both human and mouse embryogenesis [4]. IMP3 is regarded as a novel oncofetal protein that can be re-expressed in a lot of malignant tissues, including pancreatic, lung, kidney and ovarian cancers et al [5–8]. The expression of IMP3 was identified to correlate with tumor aggressive progression, suggesting that IMP3 may play a role in tumor invasion and metastasis [5–8]. IMP3 has been shown to be a promising predictor for RCC metastasis and poor clinical outcome in several studies [9–11], however, the mechanism of IMP3 in regulating RCC progression is almost unknown. Furthermore, the correlation of IMP3 expression with the clinicopathological parameters in localized CCRCC has not been fully explored. The present study was conducted to explore the molecular mechanism of IMP3 in the regulation of CCRCC progression and validate the prognostic significance of IMP3 in patients with localized CCRCC in a large cohort. We have demonstrated that IMP3 significantly promoted CCRCC cell migration and invasion via a mechanism by which IMP3 activates NF-κB pathway. NF-kB, being a well-known important transcription factor involved in cell proliferation, development, and tumorgenesis, has identified to be constitutively active in many human solid tumors including RCC [12, 13]. There are emerging studies suggest that NF-kB plays a pivotal role in the development, progression, invasion and metastases of RCC [14, 15]. A subset of NF—κB regulators and targets are shown to be upregulated in RCC and may correlate with the poor prognosis and survival [13]. The possible association of IMP3 and NF-κB is deserve further exploration.

Furthermore, we found that IMP3 expression was significantly associated with the stage and survival of localized CCRCC patients using tissue microarray, indicating that IMP3 is involved in CCRCC progression. These findings suggest that IMP3 may promote RCC progression through activating NF-κB pathway and shed new light on the elucidation of the mechanism of IMP3 in RCC progression.

## Materials and Methods

### Cell culture and reagent

Human renal carcinoma cell lines (Caki-1, Achn, 786-o, 769-p, A498) and normal human renal tubular epithelial cells HKC were obtained from the Cell Type Collection Center of the Institute of Basic Medicine, Chinese academy of medical sciences (Beijing, China). The catalogue numbers of these cell lines are listed in S1 Table. 786-o and 769-p cells were cultured in RPMI 1640 medium (Hyclone) with 10% FBS (Gibco). HKC cells were cultured in DMEM/F12 (HyClone) medium with 10% FBS, added with 100 U/ml penicillin and 100 U/ml streptomycin (Invitrogen). Caki-1 cells were cultured in HAM’S/F-12 medium with 10% FBS, Caki-1-con and Caki-1-IMP3 were grown in above medium with 5μg/ml Blasticidin (Invivogen). Achn and A498 cells were cultured in minimum essential medium (MEM; HyClone) with 10% FBS, Achn-con shRNA and Achn-IMP3shRNA cells were grown in above medium with 300 μg/ml neomycin G418 (Invitrogen). Growth media were changed every other day. Mouse anti-β-actin antibody was bought from Zhongshan (Guangzhou, China). Rabbit anti-P50, P52, P65 and IκB-α phosphorylated at S32+S36 were purchased from Bioworld (Nanjing, China). NF-κB pathway inhibitor (BAY 11–7082) was bought from Sigma (Sigma-Aldrich).

### Transfection and establishment of stable cell lines

IMP3 cDNA (TrueClone Full-Length cDNA clone, Origene) was amplified by PCR, inserted in the XhoI and Sac II sites of pLenti6/V5 plasmid, and transfected to the 293T cells to obtain the virus. Then the Caki-1 cells were transduced with the virus. Two days post-transduction, cells were cultured in selection medium with 5 μg/ml blasticidin until untransducted cells died.

Achn cells were transfected with control shRNA or IMP3 shRNA plasmids separately. The vector structures were described by An et al [16], the sequence of IMP3 shRNA was listed in S2 Table. For transfection, cells were plated in 6-well plates (1.5 ×10^5^ cells/well) 24 h before and transfected with Lipofectamine 2000 (Roche Applied Science) according to the manufacturer’s instructions. Two days post-transfection, cells were cultured in selective medium with the addition of 800 μg/ml Geneticin (Invitrogen) until untransfected cells died.

### Western blot analysis

Cell lysates were prepared using PBSTDS lysis buffer containing 1× cocktail inhibitor (Boehringer). Samples were heated at 95°C for 5 min and then separated on SDS-PAGE gels. Membranes were immunoblotted with indicated primary antibodies overnight at 4°C. After extensive washing in TBS buffer, the membranes were incubated with HRP-conjugated secondary antibody for 1 h at room temperature. Immobilized antibodies were then detected by enhanced chemiluminescence (Amersham Biosciences).

### Real-time quantitative PCR

Total RNA from cells was extracted by Trizol (Invitrogen) and quantified. According to the manufacturer’s protocol and the concentration was determined spectrophotometrically at A260. 2 μg total RNAs were used for reverse transcription using MMLV Reverse Transcriptase (Promega). Real-time qPCR was carried out using SYBR Green mix (Applied Biosystems) with PCR condition: 95°C 3 min; 95°C 20 s, 60°C 1 min, for 35 cycles. The sequences of the primer pairs are given in S3 Table. Expression of genes was determined by the comparative CT method (2^-ΔΔct^). All genes were normalized to GAPDH levels. Quantitative PCR were analyzed in triplicate and the experiments were repeated for three times.

### RNA interference

Three sequences targeting IMP3 and control siRNA were purchased from Ruibo (Guangzhou, China). The sequences of siRNAs are listed in S4 Table. Both IMP3 siRNAs and control siRNA were used at final concentration of 25 μM. Achn cells were maintained with transfection medium for 24 h, then the medium was replaced with MEM containing 10% FBS.

### Cell migration and invasion

Assays were performed using Transwell chambers (8-μm polycarbonate membrane, Costar, Corning Inc) that had been coated with or without Matrigel (BD Biosciences, Billerica) for migration and invasion assays separately.

Cells were harvested and adjusted to 5×10^5^/ml using adhesion buffer. 100 μl cells were added to the upper chamber. For migration assay, lower chamber was coated with 10 μg/ml collagen. After 8–10 h, cells attached to the filter were fixed with methanol and then stained with crystal violet (0.1%). For invasion assay, the lower chamber was loaded with NIH3T3 medium. After 24–48 h of incubation, the non-invading cells on the upper side of the chamber were removed. The membranes were fixed with methanol, and stained with Crystal violet. The number of migration and invasion cells was quantified by counting the number of cells in six random fields in each Transwell, and the average cell number was analyzed by Student *t*-test. All experiments were conducted in triplicate and repeated for three times.

### RNA deep sequencing

Caki-1 control and IMP3 over-expressing cells were passaged and total RNA was extracted, then the gene expression profiles were analyzed by Illumina 2000 Higseq at Biodynamic Optical Imaging Center of Peking University.

### Detection of IL-8 secretion

The Caki-1 cells were transfected with Flag or Flag-IMP3 plasmid, and Achn cells were transfected with con siRNA or IMP3 siRNA for 48 h. Then cell media were collected and IL-8 secretion was detected by ELISA (Boster, Wuhan, China).

### Patient cohort

This study was performed with the approval of Institutional Review Board (IRB 5041) of Cleveland Clinic. This study included tissue samples from 482 patients with unilateral, sporadic localized CCRCC who underwent radical or partial nephrectomy between January 1990 and December 2003 from Cleveland Clinic (Cleveland, Ohio, USA). Of note, patients presenting metastases at the initial diagnosis were excluded. For each patient, comprehensive clinical, pathological and outcome data elements were recorded. Tumor grade was determined using the Fuhrman grading system. Tumor necrosis was defined as microscopic coagulative necrosis. Pathological stage was reassigned according to the 2010 American Joint Committee on Cancer TNM classification. A dedicated urological pathologist (Aydin Hakan) reviewed all the cases to confirm the diagnoses.

The patients were predominantly male (62%) with a median age of 61 years (range, 23–85 years). Forty-three percent of patients had partial nephrectomies and 57% had radical nephrectomies. Most patients had low stage (T1, 67%) and low grade (Fuhrman grade 1, 51%) tumors. Necrosis was present in 19% of tumors.

### Tissue microarray (TMA) construction

Archived formalin-fixed, paraffin-embedded tumor specimens from the cohort of 482 patients were used for TMA construction. Three 1.5 mm cores were taken from at least one representative tumor block from each case and arrayed using a custom-built instrument. Tumor adjacent to necrotic tissue was avoided. Additional 3 cores were taken from the adjacent normal kidney tissue from 75 specimens.

### IMP-3 immunohistochemical (IHC) stain and evaluation

IHC staining on TMA slides was performed on the Discovery XT automated stainer (Ventana Medical Systems) using standard procedures. The tissue sections were incubated with a monoclonal antibody against IMP3 (1:100, L523S; Dako) at 4°C overnight. Negative controls were done by replacing the primary antibody with nonimmune IgG.

IMP3 expression was recorded as negative or positive after visual assessment by a genitourinary pathologist (Huiying He) without prior knowledge of patient outcome. Positive staining of IMP3 was defined as dark brown cytoplasmic staining pattern in the tumor cells, which can be easily observed at low-power (4X objective lens) magnification. Scant fine granular background staining of epithelial cells, which cannot be seen at low-power magnification or no staining was considered negative.

### Statistical analysis

The association between IMP3 expression and the tumor clinicopathologic parameters was analyzed by Fisher’s exact test for categorical variables with 2 levels; Cochran-Armitage trend test for categorical factors with >2 levels; and Wilcoxon rank sum test for measured variables. Kaplan-Meier curves were used to observe the associations of IMP3 expression with clinical outcomes. Recurrence-free survival was defined as the interval from diagnosis to documented recurrence, while overall survival was measured from diagnosis to death or last contact. Patients who had not recurred or who died without evidence of recurrence were censored at their last cancer assessment. The magnitudes of these associations were evaluated using Cox proportional hazards regression models and summarized with hazard ratios and their 95% confidence intervals (CI). The significance of the interactions was tested by Wald test. Statistical analyses were performed using the SAS 9.2 software package (SAS Institute). All tests were 2-sided and *p*<0.05 was considered statistically significant.

## Results

### IMP3 promotes cell migration and invasion in RCC cells

As previous studies showed, IMP3 protein expression was significantly associated with RCC metastasis. We speculated that IMP3 may play a role in the invasion of RCC cells. First, the expression of IMP3 in RCC cell lines and HKC cells (normal human renal epithelial Cells) were examined. As shown in Fig 1. 1A, IMP3 expression was increased in RCC cell lines compared to HKC cells. In addition, Caki-1 cells stably expressing IMP3 by retroviral transduction and Achn cells with stable knockdown of IMP3 were established (Fig 1B and 1C). We then assessed the effect of IMP3 on cell migration and invasion by Transwell assays. Overexpression of IMP3 in Caki-1 cells significantly promoted cell migration and invasion (Fig 2A and 2C). In comparison, both stable depletion of IMP3 by shRNA (Fig 2B and 2D) and transient knockdown of IMP3 by siRNA (Fig 2E and 2F) inhibited the migration and invasion of Achn cells. To rule out the possibility that the effect of IMP3 on migration is caused by cell proliferation, we knocked down IMP3 and found that depletion of IMP3 did not affect cell proliferation (S1 Fig). These data demonstrated that IMP3 could promote the migration and invasion of RCC cells.

**Fig 1:** Establishment of stable cell lines with IMP3 overexpression or knockdown. Expression of IMP3 in a panel of RCC cell lines and normal HKC cells by Western blot analysis (A). Stable overexpression of IMP3 in Caki-1 cells (left panel) transfected with FLAG-IMP3 vector and knockdown of IMP3 in Achn cells (right panel) by ShRNA (B). Real time-qPCR was performed to detect the relative mRNA expression of IMP3 in IMP3 overexpression or knockdown cells (C). Values shown are mean ± SEM of three independent experiments. * *p*< 0.05 *vs*. control group.

**Fig 2:** IMP3 promotes RCC cell migration and invasion. Transwell migration and invasion assays were used to detect the migration and invasion ability of RCC cells with IMP3 stable overexpression or knockdown. Migration of RCC cells with stable IMP3 overexpression or knockdown was measured. Caki-1-con and Caki-1-IMP3 cells (A), Achn-con shRNA and Achn-IMP3 shRNA cells, * *p*<0.0001 (B). Invasion of RCC cells with stable IMP3 overexpression or knockdown was measured. Caki-1-con and Caki-1-IMP3 cells, * *p*<0.0001 (C). Achn-con shRNA and Achn-IMP3 hRNA cells, * *p*<0.05 (D). Achn cells were transfected with control siRNA or IMP3 siRNA for 48 h and then the migration (E) and invasion (F) were detected. Values shown are mean ± SEM of three independent experiments. * *p*<0.05 *vs*. control group.

### Enhanced expression of IMP3 activates NF-κB pathway in RCC cells

To elucidate the mechanisms by which IMP3 promotes tumor cell invasion, we compared the gene expression profiles of Caki-1 overexpressing IMP3 and control cells by RNA sequencing. The entire RNA sequencing data was enclosed in S5 Table. We found that the expression of many genes involved in cell-extracellular matrix (ECM) adhesion, angiogenesis were obviously upregulated in IMP3 overexpressing cells, while the expression of some genes involved in cell-cell adhesion were down-regulated. Interestingly, 11 of NF-κB activated signature genes were found to be upregulated in IMP3 overexpressing Caki-1 cells (Fig 3A and 3B, S6 Table), suggesting that overexpression of IMP3 may activate NF-κB signaling pathway. To confirm the RNA sequencing results, the expression of some selected genes was analyzed by Real-time qPCR (Fig 3C) and found to be in agreement with the RNA sequencing data. We also found that the expression of a group member of CXC-chemokine family including IL-8, IL-6 and CCL20 together with interleukins were upregulated. It was known that IL-8 is an important downstream player in the NF-κB pathway. As shown in Fig 3D and 3E, overexpression of IMP3 increased the secretion of IL-8 in Caki-1 cells, whereas knockdown of IMP3 in Achn cells inhibited the secretion of IL-8. In addition, two other members of NF-κB family, i.e. p50 and p52, were upregulated in IMP3 overexpressing Caki-1 cells. We continued to detect the expression of NF-κB family members including p50, p52, p65, RelB and C-Rel in IMP3 overexpressing Caki-1 cells and in IMP3 depleted Achn cells. The expression of p50 and RelB was elevated in Caki-1 cells stably overexpressing IMP3 in total cellular (Fig 3F) and nuclear protein extracts (Fig 3G), and was reduced in IMP3 depleting Achn cells. At the same time, the expressions of p52, p65 and c-Rel were not affected significantly by stable overexpression or depletion of IMP3 (S2 Fig). However, transient knockdown of IMP3 by siRNA decreased the expression of p65 in Achn cells. (Fig 3H). Furthermore, we found that the phosphorylation of IkBα, the most abundant inhibitory molecule of NF-κB, was reduced by IMP3 depletion (Fig 3I). These findings suggested IMP3 activates NF-κB signaling pathway.

**Fig 3:** IMP3 overexpression activates NF-κB signaling pathway in CCRCC cells. Genes involved in adhesion, angiogenesis, chemotactic factors and interleukins in IMP3 overexpressed Caki-1 cells were showed in heat maps (A). NF-κB pathway active signature genes were upregulated in IMP3 overexpressed Caki-1 cells by RNA sequencing (B). Relative mRNA expression of cytokines was detected by real-time PCR in IMP3 overexpressed Caki-1 cells (C). The Caki-1 cells were transfected with Flag-IMP3 vector. Forty eight hoursh after transfection, the culture medium was removed and added with serum free medium for 24 h, the medium was harvested. The secretion of IL-8 was detected by ELISA. Values are means ± SD of three independent experiments. * p<0.05 vs. empty vector (D). The Achn cells were transfected with IMP3 siRNA or control siRNA. The identical management was given to cells as shown in D. * p<0.05 vs. control (E). Western blot analyses of P50 and RelB expression in total protein (F) and nuclear extracts (G) in IMP3 overexpressed Caki-1 cells and Achn knockdown cells. Actin and YY1 were used to control the loading. The Caki-1 cells were transfected with Flag-IMP3 vector. The Achn cells were transfected with IMP3 siRNA or control siRNA. Forty eight hours after transfection cells were harvested, the expression of P65 (H) and p-IκBα (I) was detected by Western blot.

### IMP3 promotes cell motility through NF-κB pathway in RCC

To determine whether IMP3 promoted the motility of CCRCC cells through NF-κB pathway, BAY 11–7082 (a specific IKK inhibitor) was used to inhibit the activation of NF-κB pathway. Our results showed that the migration-promoting effect of IMP3 was inhibited by BAY 11–7082 in Caki-1 cells (Fig 4A and 4B). Furthermore, as shown in Fig 4C, BAY 11–7082 significantly inhibited IMP3- induced phosphorylation of IκBα (Fig 4C). These results suggested that IMP3 may promote cell migration through NF-κB pathway.

**Fig 4:** IMP3 promotes RCC cell migration through NF-κB pathway. Caki-1 cells were transfected with FLAG or FLAG-IMP3 vector for 48 h followed by treatment with or without BAY 11–7082 (20 μM) for 1h, and then cells were harvested for Transwell or Western blot assays. Transwell migration assay was used to detect the migration of RCC cells with IMP3 overexpression. Values shown are mean ± SEM of three independent experiments. * *p*<0.05 (A-B). The expression of P-IκBα was detected by Western blot (C).

### IMP3 is an independent prognostic biomarker for localized CCRCC

Four hundred and sixty nine cases of localized CCRCC were finally assessed for IMP3 expression with 13 cases eliminated due to insufficient tissues after IHC staining. Overall, sixteen percent (73/469) of tumors stained positive for IMP3 (Fig 5A and 5B). No expression of IMP3 was detected in the benign kidney tissue adjacent to the tumors.

**Fig 5:** IMP3 expression in localized clear cell renal cell carcinoma and Kaplan-Meier survival analyses. A-B: Representative IMP3 immunostaining: negative (A, n = 299), positive (B, n = 48) immunoreactivity in localized CCRCC on tissue array. C-D: Kaplan-Meier survival analyses of CCRCC patients. Correlation of negative (n = 299) and positive IMP3 expression (n = 48) with recurrence free survival (C) and overall survival (D) were analyzed by univariate survival analysis (*p*<0.0001).

IMP3 expression was found significantly associated with all the examined pathological parameters, including tumor size, nuclear grade, tumor stage, perinephric fat invasion, necrosis and sarcomatoid element (*p*<0.0001, Table 1). Only 25% of stages I and II tumors expressed IMP3, whereas 58% of stages III and IV tumors expressed this protein. IMP3 was expressed mainly in high-grade (69%, grades 3 and 4) tumors versus low-grade tumors (7%, grades 1 and 2). IMP3 positivity was significantly increased in patients with sarcomatoid element (65%). Univariable analysis of recurrence-free survival and overall survival is showed in S7 and S8 Tables.

**Table 1:** Association between the clinicopathological parameters and IMP3 expression.

Factor		IMP3(-)	IMP3(+)	*p* ^1^	overall
Gender^2^					
	Male	181 (83%)	37 (17%)		218 (62%)
	Female	120 (92%)	11 (8%)	***0*.*03***	131 (38%)
Age^2^					
	Mean ± s.d.	60 ± 11.9	64 ± 9.8		60 ± 11.7
	Median	61	64		61
	Range	23–85	48–83	***0*.*05***	23–85
Nuclear Grade (Fuhrman)^3^					
	1,2	222 (93%)	16 (7%)		238 (51%)
	3	150 (82%)	32 (18%)		182 (39%)
	4	23 (49%)	24 (51%)	***<0*.*0001***	47 (10%)
Perinephric Fat Invasion^3^					
	No	356 (87%)	51 (13%)		407 (87%)
	Yes	39 (65%)	21 (35%)	***<0*.*0001***	60 (13%)
Microscopic Vascular Invasion^3^					
	No	339 (88%)	45 (12%)		384 (82%)
	Yes	56 (67%)	27 (33%)	***<0*.*0001***	83 (18%)
T-Stage^4^					
	T1	281 (90%)	30 (10%)		311 (67%)
	T2	33 (85%)	6 (15%)		39 (8%)
	T3a	33 (72%)	13 (28%)		46 (10%)
	T3b, T3c	49 (70%)	21 (30%)	***<0*.*0001***	70 (15%)
Tumor Size (cm)^4^					
	Mean ± s.d.	4.9 ± 3.0	7.3 ± 4.2		5.3 ± 3.3
	Median	4	6		4.5
	Range	1.0–17.0	1.3–20.5	***<0*.*0001***	1.0–20.5
Necrosis^5^					
	No	342 (90%)	38 (10%)		380 (81%)
	Yes	54 (62%)	34 (39%)	***<0*.*0001***	88 (19%)
% Necrosis (when present)					
	Mean ± s.d.	8.2 ± 10.6	14.7 ± 15.7		10.7 ± 13.1
	Median	3	8.1		5
	Range	0.3–43.0	0.5–75.7	***0*.*008***	0.3–75.7
Sarcomatoid Element^5^					
	No	389 (87%)	59 (13%)		448 (96%)
	Yes	7 (35%)	13 (65%)	***<0*.*0001***	20 (4%)
% Sarcomatoid (when present)					
	Mean ± s.d.	13.8 ± 21.7	4.3 ± 6.1		7.6 ± 13.9
	Median	4	1.1		1.6
	Range	1.0–60.0	0.2–18.3	**0.*14***	0.2–60.0

^1^ Fisher’s exact test for categorical variables with 2 levels; Cochran-Armitage trend test for categorical factors with >2 levels; and Wilcoxon rank sum test for measured variables.

^2^ Missing for 120 patients

^3^ Missing for 2 patients

^4^ Missing for 3 patients

^5^ Missing for 1 patient

Three hundred and forty seven patients were included in the survival analysis. Expression of IMP3 correlated with short survival of localized CCRCC patients (Fig 5C and 5D). Patients with IMP3-negative tumors had significantly longer recurrence-free survival and overall survival than those with IMP3 positive tumors. Five-year recurrence-free survival was 87% ± 2% in patients with IMP3-negative tumors versus 48% ± 8% (*p*<0.0001) in those with IMP3-positive tumors (Fig 5C). Five-year overall survival was 87% ± 2% in patients whose tumors did not express IMP3 versus 52% ± 7% (*p*<0.0001) in those whose tumors did express IMP3 (Fig 5D). The hazard ratio of IMP3 expression was 4.51 for recurrence-free survival and 3.63 for overall survival (S7 and S8 Tables).

Multivariable analysis of recurrence-free and overall survival is summarized in Table 2. Positive IMP3 staining, tumor necrosis and perinephric fat invasion were all independent prognostic factors for both recurrence-free and overall survival of localized CCRCC. Taken together, IMP3 was validated to be an independent prognostic factor for localized CCRCC patients, and patients with IMP3 positive tumors have a shorter survival than those with IMP3 negative tumors.

**Table 2:** Multivariable analyses of prognostic factors for localized CCRCC.

**A. Time to Recurrence (n = 344)**			
**Factor b** ± **s.e.**		**Hazard Ratio (95% C.I.)**	***P***
IMP3 Staining Intensity (>0 vs 0)	1.02 + 0.26	2.78 (1.67–4.60)	<0.0001
Perinephric Fat Invasion (Yes vs No)	1.16 ± 0.29	3.21 (1.81–5.70)	<0.0001
Necrosis (Yes vs No)	1.19 ± 0.28	3.30 (1.91–5.70)	<0.0001
Tumor size (per cm)^1^	0.13 ± 0.05	1.14 (1.04–1.25)	0.005
**B. Survival (n = 346)**			
**Factor b** ± **s.e.**		**Hazard Ratio (95% C.I.)**	***P***
IMP3 Staining Intensity (>0 vs 0)	0.80 ± 0.23	2.22 (1.41–3.50)	0.0006
Necrosis (Yes vs No)	0.71 ± 0.25	2.03 (1.24–3.32)	0.005
Perinephric Fat Invasion (Yes vs No)	0.68 ± 0.27	1.97 (1.16–3.35)	0.01
Nuclear Grade (3,4 vs 2 vs 1)	0.45 ± 0.18	1.57 (1.10–2.25)	0.01

Wald test from proportional hazards model

^1^ Larger tumors is associated with poorer outcome; tumors >10 cm were combined into a single group.

## Discussion

CCRCC is the most aggressive subtype of common RCC and it is lethal when metastatic [17, 18]. IMP3 was identified to be a promising biomarker for metastatic RCC [19], however, the possible mechanism of IMP3 regulating RCC progression is largely unknown. Furthermore, it is important to develop prognostic markers for localized CCRCC. IMP3 has been suggested to be a valuable prognostic marker for metastatic and localized CCRCC in a few studies. The prognostic and risk stratified value of IMP3 in localized CCRCC is required to be validated. In the present investigation, we identified a novel mechanism that IMP3 controls RCC progression by promoting RCC cell migration and invasion via activation of NF-κB pathway. In addition, we validated the use of IMP3 as a prognostic marker for localized CCRCC. Although numerous descriptive studies suggested that IMP3 expression correlates with tumor aggressiveness in a variety of malignancies [8, 20–23], the role of IMP3 in modulating tumor cellular functions was poorly understood. To our knowledge so far there was no report on mechanisms underlying IMP3 regulation of RCC progression. Our data showed that IMP3 promotes RCC cell migration and invasion, which was consistent with previous findings of IMP3 in breast carcinoma [24]. The EGFR signaling pathway was shown to regulate the expression of IMP3 and is involved in IMP3 promotion of breast cancer cell migration and invasion by up-regulation of CD164 and matrix metalloproteinase 9 (MMP9) [24]. However, we did not demonstrate EGF regulation on IMP3 expression in Caki-1 cells (unpublished data), suggesting that IMP3 in RCC may not function through EGFR signaling pathway. Intriguingly, we identified that IMP3 activates NF-κB pathway in RCC cells and IMP3 promotes RCC cell migration through NF-κB pathway. The NF-κB family consists of five members: RelA (p65), RelB, c-Rel, NF-κB1 (p105/p50) and NF-κB2 (p100/p52). The NF-κB pathway was reported to be involved in almost all important aspects of RCC progression including angiogenesis, invasion, metastasis and multi-drug resistance [14]. By immunostaining of p50 and p65, there was a study suggesting a correlation between invasion and metastasis of RCC and the expression and activation of NF-κB [15]. However, the relationship between IMP3 and NF-κB was not established. By analyzing the gene expression profile of IMP3 overexpressed RCC cells using RNA deep sequencing, we demonstrated for the first time that the genes involved in NF-κB signaling pathway including p50 and RelB were indeed upregulated by IMP3.

Normally, NF-κB is sequestered in the cytoplasm in an inactive form, and bound to one of many inhibitory molecules (IκBs), of which IκBα is the most abundant one. IκBα forms a complex with P50/P65, making an inactive complex in cytoplasm. The phosphorylation of IκBα leads to the active NF-κB being translocated to the nucleus where it binds to κB sites on target genes and induces the transcription of oncogenes that regulate apoptosis, angiogenesis, invasion, metastasis and multi-drug resistance [14]. Our data showed that overexpression of IMP3 increased phosphorylation of IκBα and knockdown of IMP3 reduced activation of IκBα in RCC cells, indicating further that IMP3 activates the NF-κB signaling pathway.

NF-κB controls cell migration and invasion via transcriptional activation of downstream pro-migratory and pro-invasive genes including CXC chemokines, urokinase-type plasminogen activator and MMPs [25]. Chemokines and chemokine receptors appear to play an integral role in survival, growth, and metastasis of RCC [26]. IL-8, also known as CXCL-8, is a potent pro-inflammatory cytokine that belongs to the CXC chemokine family of proteins. In addition to its pro-inflammatory role, IL-8 is also known to play an important role in angiogenesis, tumor growth and metastasis of multiple cancers including RCC [27–29]. In this study, we found that overexpression of IMP3 increased the secretion of IL-8 and IL-8 secretion was reduced after knockdown of IMP3 in RCC cells. We also found that other CXC chemokines such as IL-6 and CCL20 were upregulated in IMP3 overexpression cells by RNA-sequencing and real-time PCR. Furthermore, our results suggested that IMP3-promoted cell migration could be inhibited by NF-κB pathway inhibitor, indicating that IMP3 promoting RCC cell migration requires activation of NF-κB pathway, which represents a novel mechanism accounting for IMP3 regulation of cancer progression. Although IMP3 has been known to be associated with distinct cancer types, the functional role of IMP3 is barely investigated. Only a few target mRNAs and some putative candidates are identified. IGF2 is validated as a key target transcript of IMP3. In the present study, the level of IGF2 mRNA was shown to be significantly upregulated by IMP3 overexpression (our RNA sequencing data in S5 Table). IGF-II was shown to induce steroid sulfatase expression via a PI3-kinase/Akt-NF-κB signaling pathway in PC-3 cells and may induce estrogen-mediated carcinogenesis [30]. However, whether IMP3 regulation of NF-κB signaling pathway is mediated by IGF2 warrants future investigations.

Another important finding we made in this study is that IMP3 is validated as an independent prognostic marker for localized CCRCC, which is concluded based on comprehensive analyses of our large cohort of localized CCRCC patients. IMP3 was also found to be associated with several recognized clinicopathological variables including Fuhrman nuclear grade, pathological T-stage, sarcomatoid differentiation and coagulative necrosis. IMP3 expression can improve risk stratification for localized CCRCC patients and it may become a novel therapeutic target for patients with high risk CCRCC. Several studies showed that IMP1 and IMP3 may function collaboratively and were the prognostic markers of various types of cancer including breast, ovarian, melanoma and colon cancers [22, 31–33]. No indication of IMP1 expression in RCC was reported. In a separate study, we detected IMP1 expression in 28% of localized CCRCC (130/469) and found that there was no correlation between IMP1 and IMP3 expression. In addition, the expression of IMP1 did not associate with any clinicopathological characteristics of CCRCC (unpublished data).

In summary, we found that IMP3 regulates RCC cell migration and invasion through activation of NF-κB signaling pathway. A series of chemokines, especially IL-8, may have important roles in IMP3 promoting the RCC cell progression. IMP3 is validated to be an independent prognostic marker for localized CCRCC. Therefore, IMP3 may represent a novel therapeutic target for RCC patients.

## Supporting Information

S1 Fig IMP3 knockdown did not affect the proliferation of ACHN cells. The WST1 assay was performed to examine the proliferation of ACHN-IMP3sh and control cells. The cells were seeded into 96-well plates, and the absorbance at 490 nm was measured at the indicated time points.
(TIF)

S2 Fig The C-Rel, P65 and P52 expression of NF-kB was not influenced significantly by IMP3 overexpression or knockdown. Western blot analyses of C-Rel, P65 and P52 expression in total protein (A) and nuclear extracts (B) in IMP3 overexpressed Caki-1 cells and Achn knockdown cells. Actin and YY1 were used to control the loading. The Caki-1 cells were transfected with Flag-IMP3 vector. The Achn cells were transfected with IMP3 siRNA or control siRNA. Forty eight hours after transfection cells were harvested, the expression of C-Rel, P65 and P52 was detected by Western blot.
(TIF)

S1 File Supporting information containing individual subtitles for the methods and results. Our original experimental data including the transfection efficiency, the migration assay, the invasion assay, the Wst-1 assay, the real-time qPCR results, the ELISA assay and the overall survival information of the de-identified patients.
(XLS)

S1 Table The catalogue numbers of the cell lines that used in this study. (DOC)

S2 Table Sequence of IMP3 shRNA. Underlines the sense and antisense chain of IMP3 SiRNA target sequences. (DOC)

S3 Table Primers used in real-time qPCR. (DOC)

S4 Table Sequences of IMP3 siRNA. (DOC)

S5 Table RNA sequencing data of IMP3 overexpressed Caki-1 cells. (XLS)

S6 Table NF-κB pathway genes identified in IMP3 overexpressed Caki-1 cells. (DOC)

S7 Table Time to recurrence—Univariable analyses of clinicopathological parameters and IMP3 immunostaining for localized CCRCC. (DOC)

S8 Table Overall survival-Univariable analyses of clinicopathological parameters and IMP3 immunostaining for localized CCRCC. (DOC)
